# Reanalysis of the gene expression profile in chronic pancreatitis via bioinformatics methods

This article has been retracted.

**DOI:** 10.1186/2047-783X-19-31

**Published:** 2014-05-29

**Authors:** Hang Yuan, Bin Wu, Senlin Ma, Xiaoyu Yang, Lei Yin, Aijun Li

**Affiliations:** 1 Department of the 2nd Special Treatment, Eastern Hepatobiliary Surgery Hospital, Second Military Medical University, No 225, Changhai Road, Shanghai 200438, China

**Keywords:** Chronic pancreatitis, Differentially expressed genes, Gene cluster, miRNA

## Abstract

**Background:**

Diagnosis at an early stage of chronic pancreatitis (CP) is challenging. It has been reported that microRNAs (miRNAs) are increasingly found and applied as targets for the diagnosis and treatment of various cancers. However, to the best of our knowledge, few published papers have described the role of miRNAs in the diagnosis of CP.

**Method:**

We downloaded gene expression profile data from the Gene Expression Omnibus and identified differentially expressed genes (DEGs) between CP and normal samples of Harlan mice and Jackson Laboratory mice. Common DEGs were filtered out, and the semantic similarities of gene classes were calculated using the GOSemSim software package. The gene class with the highest functional consistency was selected, and then the Lists2Networks web-based system was used to analyse regulatory relationships between miRNAs and gene classes. The functional enrichment of the gene classes was assessed based on Gene Ontology (GO) and Kyoto Encyclopedia of Genes and Genomes pathway annotation terms.

**Results:**

A total of 405 common upregulated DEGs and 7 common downregulated DEGs were extracted from the two kinds of mice. Gene cluster D was selected from the common upregulated DEGs because it had the highest semantic similarity. miRNA 124a (miR-124a) was found to have a significant regulatory relationship with cluster D, and DEGs such as *CHSY1* and *ABCC4* were found to be regulated by miR-124a. The GO term of response to DNA damage stimulus and the pathway of *Escherichia coli* infection were significantly enriched in cluster D.

**Conclusion:**

DNA damage and *E. coli* infection might play important roles in CP pathogenesis. In addition, miR-124a might be a potential target for the diagnosis and treatment of CP.

## Background

Chronic pancreatitis (CP) is characterized by pancreatic inflammation and fibrosis, and it arises when pancreatic injury is followed by a sustained immune activation in which fibrosis dominates [1]. Environmental triggers of pancreatic inflammation and disease susceptibility (such as alcohol use, smoking, pancreatic duct obstruction and drugs) or modifying genes (including *PRSS1*, *SPINK1* and *CFTR*) act synergistically to cause CP [1,2]. It has also been indicated that CP is often an underlying cause of pancreatic cancer [3]. Meanwhile, in recent years, researchers in a growing number of studies have suggested that microRNAs (miRNAs) play an important role in the diagnosis and prognosis of pancreatic cancers [3-6]. miRNAs inhibit the transcription levels of mRNA, induce degradation of the regulation of gene expression [7] and have been proved to be involved in many disease processes. Therefore, the identification of miRNA changes might explain the pathology of CP in another way and provide a new method for diagnosing CP.

A number of miRNAs that have been studied have a role in pancreatic diseases. By comparing pancreatic cancer tissue to CP tissue and normal pancreas, Bloomston and colleagues identified 21 miRNAs with increased expression and 4 with decreased expression, which suggests that the miRNAs likely play an important regulatory role in pancreatic cancer [3]. It has also been demonstrated that the expression of miRNA-196a (miR-196a) is high in pancreatic ductal adenocarcinoma (PDAC) but low in CP and normal tissues, whereas miR-217 exhibits the opposite expression pattern [8]. The ratio of miR-196a to miR-217 has been found to indicate whether tissue samples contain PDAC [9]. More and more miRNAs have been found to be related to pancreatic cancers, and CP specimens are often used as a second control [3,9]. However, few published papers have specifically described the relationship between CP and its miRNAs.

In the present study, we analysed the gene expression profile of CP and normal mice to screen for differentially expressed genes (DEGs). We identified the related miRNAs, which might provide further insights into the molecular mechanisms of CP. Understanding the molecular mechanisms of CP might aid in diagnosing and treating CP patients.

## Methods

### Data sources

We downloaded a gene data set [GEO:GSE41418] [10] from the Gene Expression Omnibus (GEO) database (http://www.ncbi.nlm.nih.gov/geo/). Gene expression analysis was performed on a GeneChip Mouse Genome 430 Plus 2.0 Array platform (Affymetrix, Santa Clara, CA, USA). The data set contains two different kinds of mice: Harlan mice (C57BL/6NHsd; Harlan Laboratories, Indianapolis, IN, USA) and Jackson Laboratory mice (C56BL/6 J; The Jackson Laboratory, Bar Harbor, ME, USA). A frequently used experimental model of CP recapitulating human disease is repeated injections of cerulein into mice. We found that two common substrains of C57BL/6 mice (C56BL/6 J and C57BL/6NHsd) exhibit different degrees of CP, with C57BL/6 J mice being more susceptible to repetitive cerulean-induced CP. The goal of this study was to identify genes associated with CP and to identify differentially regulated genes between two substrains as candidates for the CP progression. We included six mice of each type, including three CP samples and three normal samples [10].

### Identification of differentially expressed genes

Expression profile data were normalized with GeneChip robust multiarray analysis [11]. Next, we preprocessed the data derived from 12 samples for subsequent analysis. We annotated expression profiling probes to gene symbols. If there were multiple probe sets that corresponded to one gene, the expression values of those probe sets were averaged. Using this method, we obtained an expression data set comprising 21,389 genes. Afterward, Significance Analysis of Microarrays 4.0 software [12] was used to screen the DEGs between the CP samples and normal controls of the two kinds of mice, respectively. The overlapping DEGs were denoted as common DEGs and were used for further analysis. A fold discovery rate (FDR) ≤0.05 was selected as the threshold for screening DEGs.

### Gene cluster analysis of common differentially expressed genes

Gene cluster analysis can be used to divide genes into several classes based on certain similarity criteria, such as the Pearson correlation coefficient or Euclidean distance [13,14]. It has been proved that genes in the same cluster have a high degree of homogeneity. In our present study, we used the second-order tolerance analysis (SOTA) method [15], a toolset of gene expression profile analysis [16], to perform cluster analysis on the common DEGs based on the gene expression values. The Euclidean distance was employed as the clustering indicator. Next, we calculated the semantic similarity of gene classes using the GOSemSim software package [17], and the class of genes with the highest functional consistency was selected as the optimal gene cluster for further study.

### Related microRNAs of optimal gene cluster and GO and KEGG pathway analysis

In organisms, highly coexpressed genes are likely to share common regulatory patterns and to participate in the same or similar biological processes and pathways [18]. In order to study the regulatory mechanisms of the optimal gene cluster, we used the Lists2Networks web-based system [19] to analyse the possible relationship between the miRNAs and the optimal gene cluster. The functional enrichment of the target genes of two regulators (transcription factors and miRNAs) was assessed based on the Gene Ontology (GO) and Kyoto Encyclopedia of Genes and Genomes (KEGG) pathway annotation terms. GO and KEGG signalling pathway analyses were performed using the GOstats R package software package (http://www.r-project.org/), with which we carried out the standard hypergeometric test. We was also performed GO and KEGG enrichment analysis on the gene cluster, with *P*-values less than 0.05 considered statistically significant.

## Results

### Identification of differentially expressed genes

According to the predetermined FDR threshold ≤0.05, 962 DEGs of Harlan mice, including 911 upregulated genes and 51 downregulated genes, were screened out. In Jackson mice, a total of 1,545 genes were differentially expressed, and these DEGs comprised 1,423 upregulated genes and 122 downregulated genes. Next, we extracted overlapping DEGs in both mice, which consisted of 405 upregulated genes and 7 downregulated genes (Figure 1). We clearly observed that the number of upregulated genes was significantly greater than that of downregulated genes. We speculate that these upregulated genes might play a major role in CP disease. In the experimental work following this observation, we analysed only the upregulated common DEGs.

**Figure 1:** **Common differentially expressed genes of the two mouse breeds studied.** The red and blue parts represent, respectively, the upregulated common differentially expressed genes (DEGs) and downregulated common DEGs.

### Gene clustering of upregulated common differentially expressed genes

Using the Euclidean distances as the clustering indicators in SOTA, we obtained four clearly separated gene classes (Figure 2) of the upregulated common DEGs. Next, we calculated the semantic similarity scores of gene classes (Table 1). As a result, gene cluster D was found to have the highest average semantic similarity score (0.2868) and was selected for further analysis.

**Figure 2:** **Dendrogram used for clustering analysis of the common upregulated differentially expressed genes.** As shown in the diagram, the genes are divided into four categories **(A**, **B**, **C** and **D)**.

**Table 1:** Semantic similarity scores of the gene clusters

**Cluster**	**Gene number**	**Semantic similarity score**
Cluster A	51	0.2145412
Cluster B	91	0.2525834
Cluster C	121	0.272545
Cluster D	110	0.2867982

### Related microRNAs and functional analysis of the optimal gene cluster

According to the enrichment analysis of Lists2Networks, miR-124a was found to have a significant regulation relationship with cluster D (Table 2). And genes such as *CHSY* (chondroitin sulphate synthase 1) and *ABCC4* (ATP-binding cassette, subfamily C (CFTR/MRP), member 4) were enriched and in correlation with miR-124a. According to GO and KEGG pathway enrichment on gene cluster D, we found that the most significant biological process was response to DNA damage stimulus (Table 3), and *PAPR3* was one of the significant DEGs enriched in the GO term. The observed significant pathways were associated with the cell cycle and *Escherichia coli* infection (Table 4).

**Table 2:** Regulatory microRNAs predicted for cluster D

**Term**	**Genes**	**Combined score**	***P*-value**
TGCCTTA, mIR-124a	*CHSY1*, *ABCC4*, *CASC4*	8.818	0.00828
TCTAGAG, mIR-517	*SLC39A10*, *RND3*	7.065	0.03707
TAGAACC, mIR-182	*FAM107B*, *RBM12*	6.138	0.02771

**Table 3:** Gene Ontology database enrichment analysis of cluster D

**Gene Ontology term**	**Genes**	***P*-value**
Response to DNA damage stimulus	*PARP3*, *TOP2A*, *RAD51*	0.0025
DNA metabolic process	*PRIM1*, *RFC1*, *PARP3*	0.0041
Chromosome organisation	*CDCA8*, *H2AFX*, *RFC1*	0.0047
Chromosome condensation	*NCAPH*, *TOP2A*	0.0065
Chromosome segregation	*MIS12*, *TOP2A*	0.0073
Cellular response to DNA damage stimulus	*TOPBP1*, *PARP3*, *TOP2A*	0.0080
mRNA export from nucleus	*AGFG1*, *RAE1*	0.0089
DNA packaging	*NCAPH*, *TOP2A*	0.0106
Response to ionizing radiation	*TOPBP1*, *H2AFX*	0.0115
RNA export from nucleus	*AGFG1*, *RAE1*	0.0124
Endocytosis	*SNX4*, *SFTPD*, *CD14*	0.0150
Regulation of ubiquitin-protein ligase activity	*BUB3*, *CDC23*, *CCNB1*	0.0155
RNA transport	*AGFG1*, *RAE1*	0.0166
DNA repair	*TOPBP1*, *PARP3*, *TOP2A*	0.0170
Nuclear export	*AGFG1*, *RAE1*	0.0290
DNA replication	*RFC1*, *TOP2A*, *MCM5*	0.0324
Organelle organisation	*CDCA8*, *BUB3*, *H2AFX*	0.0357
Response to stress	*PARP3*, *PHLDA3*, *LSP1*	0.0359
Cellular response to stimulus	*PARP3*, *TOP2A*, *RAD51*	0.0375
Innate immune response	*TUBB2C*, *SFTPD*	0.0441

**Table 4:** **KEGG enrichment analysis of cluster D**^**a**^

**KEGG_PATHWAY**	**Genes**	***P*-value**
hsa04110 cell cycle	*RBL1*, *CDC23*, *MCM5*	1.80E-04
hsa05131 enteropathogenic *E. coli* infection	*TUBB2A*, *TUBB2C*, *CD14*	0.007263
hsa05130 enteropathogenic *E. coli* infection	*TUBB2A*, *TUBB2C*, *CD14*	0.007263
hsa04115 p53 signalling pathway	*CCNB1*, *CCNB2*, *APAF1*	0.013926
hsa04640 hematopoietic cell lineage	*CD38*, *IL1R1*, *CD14*	0.026877
hsa00600 sphingolipid metabolism	*SGMS1*, *B4GALT6*	0.034673

^a^*E. coli*, *Escherichia coli*; KEGG, Kyoto Encyclopedia of Genes and Genomes.

## Discussion

In the present study, we screened out 405 common upregulated DEGs of the two kinds of mice used, and GOSemSim was used to calculate the semantic similarity of the gene clusters of the DEGs. Cluster D was selected as the optimal gene class for further investigation because of it had the highest average semantic similarity. Using the Lists2Networks, we found that cluster D could be significantly regulated by miR-124a, which might play an important role in the development of CP.

miR-124a was first identified by cloning studies in mice [20]. Studies have shown that miR-124a plays an important role in the control of cell survival, proliferation, differentiation and metabolism and whose dysfunction is a potential cause of disease [21-23]. In addition, published data have demonstrated that miR-124a expression level was increased in the mouse pancreas at the embryonic stage and have indicated its important role in pancreas development [23]. Therefore, we hypothesized miR-124a might play an important pathogenic role in CP.

*CHSY1* encodes a member of the chondroitin *N*-acetylgalactosaminyltransferase family, possesses dual glucuronyltransferase and galactosaminyltransferase activity and plays critical roles in the biosynthesis of chondroitin sulphate, a glycosaminoglycan involved in many biological processes, including cell proliferation and morphogenesis [24-26]. *CHSY1* was one of the significant genes in cluster D and was enriched and regulated by miR-124a. Researchers in a previous study demonstrated that *CHSY1* regulated its downstream target *CASP1* (caspase 1, also known as interleukin 1β–converting enzyme), which could cleave interleukin 1β precursors into mature cytokines and contribute to inflammation [27]. Surprisingly, increased expression of CASP1 has been reported to be a frequent event in CP [28]. Thus, miR-124a might participate in CP manifestation and development by regulating expression levels of *CHSY1* or *CASP1*.

*ABCC4* is another significant gene regulated by miR-124a. It is a member of the ATP-binding cassette transporter superfamily, which has been shown to comprise key mediators of drug efflux and multidrug resistance in many types of tumours and inflammatory diseases [29-31]. A previous study also been implicated ABCC4 as an efflux pump of proinflammatory mediators such as LTB4 and LTC4, and ABCC4 may represent a novel target for anti-inflammatory therapies [32]. Therefore, miR-124a might regulate the inflammatory disease of CP by changing the levels of proinflammatory mediators by ABCC4.

On the basis of the results of GO enrichment analysis of gene cluster D, the most significant biological process we observed was the response to DNA damage stimulus. This suggested that DNA damage might play an important role in the pathogenesis of CP. The results of our analysis are in line with those of a previous study [33]. *PARP3* is one significant gene that is enriched in the biological process of response to DNA damage stimulus. It belongs to the poly(ADP-ribose) polymerase (PARP) family [34]. *PARP3* catalyses the reaction of ADP ribosylation, a key posttranslational modification of proteins involved in different signalling pathways from DNA damage to energy metabolism and organismal memory [35]. In addition, recent studies have clearly demonstrated the role of PARP activation in various forms of local inflammation [36-38]. Information about the role of *PARP3* in CP is sparse; however, it has been shown that other members of the PARP family, such as PARP1, coactivate the transcription factor nuclear factor κB (NF-κB) and is required for NF-κB-mediated inflammatory responses [39]. CP is characterized by pancreatic inflammation, thus *PARP3* might potentially play a role in its inflammatory processes.

In KEGG pathway analysis, it has been shown that *E. coli* infection might play an important role in CP. Karmali and colleagues reported that infection with *E. coli* produced postdiarrhoeal haemolytic uraemia syndrome and that many patients who recovered from it had long-term sequelae, including CP and cholelithiasis [40,41]. Furthermore, *E. coli* might also lead to pancreatic abscess, which is defined as an acute inflammatory process of the pancreas [42]. It has been proved that *E. coli* organisms can induce polymorphonuclear leucocyte infiltration during clinical infection [43]. Therefore, we suggest that *E. coli* infection might be involved in the occurrence of CP.

This study has some limitations. First is the small sample size obtained from the GEO database. Second, validation of the results in other data sets or samples is lacking. Therefore, further genetic studies with larger sample sizes and different kinds of CP samples are needed to confirm our observations.

## Conclusions

miR-124a provides some guidance for the mechanism of CP pathogenesis and is a potential target for the diagnosis and treatment of CP. miR-124a might participate in CP occurrence and development by regulating expression levels of CHSY1 or CASP1. Also, miR-124a might regulate the inflammatory disease of CP by changing the level of proinflammatory mediators by ABCC4. In addition, DNA damage and *E. coli* infection might play important roles in CP pathogenesis.

## Abbreviations

CASP1: Caspase 1, also known as interleukin-1β-converting enzyme; CP: Chronic pancreatitis; DEG: Differentially expressed gene; GEO: Gene Expression Omnibus; GO: Gene Ontology; KEGG: Kyoto Encyclopedia of Genes and Genomes; PARP: Poly(ADP-ribose) polymerase; PDAC: Pancreatic ductal adenocarcinoma; SAM4.0: Significance Analysis of Microarrays 4.0 software; SOTA: Second-order tolerance analysis.

## Competing interests

The authors declare that they have no competing interests.

## Authors’ contributions

YH and LAJ carried out the molecular genetic studies, participated in the sequence alignment and drafted the manuscript. YH carried out the immunoassays with WB participated in the sequence alignment. WB and MSL participated in the design of the study and performed the statistical analysis. YXL and YL conceived of the study, and participated in its design and coordination and helped to draft the manuscript. All authors read and approved the final manuscript.

## Authors’ information

HY and BW should be regarded as co–first authors.
